The article "Effects of Personality Characteristics of Different Genders and Quality of Life Analysis on Risk Factors for Suicide in Depressive Patients" was published in 2021. Journal: Comput Math Methods Med.

# Effects of Personality Characteristics of Different Genders and Quality of Life Analysis on Risk Factors for Suicide in Depressive Patients

**DOI:** 10.1155/2021/7850281

**Published:** 2021-12-18

**Authors:** Xuebing Xu, Jing Jiang, Hongjuan Bai, Tao Tian

**Affiliations:** Ningxia Ning-An Hospital, 236 Jinbo South Street, Xixia District, Yinchuan, Ningxia 750021, China

## Abstract

**Objective:**

The study was to explore the roles of personality characteristics of different genders and analyze the risk factors of quality of life (QOL) analysis in suicide among depressive patients.

**Methods:**

One hundred and eighty-six depressive patients from January 2018 to March 2019 in the Department of Psychiatry of our hospital were enrolled and divided into Groups A and B considering whether they had a suicidal tendency or not. Among them, 90 in Group A had a suicidal tendency and consisted of 42 males and 48 females, while 96 in Group B had no suicidal tendency and consisted of 44 males and 52 females. Forward and backward selection and then backward selection were performed on all the variables of gender characteristic factors and QOL factors that may cause suicide, on which stepwise regression was finally conducted. Next, univariate logistic regression analysis was first performed to select important variables from the related risk factors that may cause suicide, and then, the multivariate logistic regression model was used to select important independent risk factors. *Results and Conclusion*. The age of onset, degree of anxiety, moral support, positive mental attitude, and family independence were the independent risk factors that may cause a suicidal tendency for male depressive patients. The age of onset, degree of anxiety, negative life events, moral support, positive mental attitude, family intimacy, psychoticism, and neuroticism were the independent risk factors for female depressive patients. Physiological function, role physical, bodily pain, social function, and emotional role in QOL may be the independent risk factors for a suicidal tendency.

## 1. Introduction

Depression, as a highly prevalent emotional disorder, is perhaps the most frequent cause of emotional suffering in later life and significantly decreases quality of life in older adults. Depression often presents with physical symptoms, primarily fatigue, pain, or sleep disturbance. Depression patients may show suicidal ideas, behaviors, and psychiatric characteristics in the worst case [1], with the lifetime prevalence of depression reported to be 7%-21% [2]. Depression is not a normal part of the aging process. Common among patients seeking treatment in primary health care institutions, the disease is the major cause of disability for people aged 15 and over, and it affects individuals, families, businesses, and society [3]. The disease is also a clinical problem that affects individuals in many different ways [4], with its lifetime prevalence among women being approximately twice that among men [5, 6]. It is estimated that 50% of depressive patients have not been treated with effective interventions. Even if they recover eventually, many of them still need trial and error, because there is no reliable guide to obtain the best treatment for them, and many of them will develop drug resistance during treatment over time [7]. In addition, the underlying pathology of depression is very heterogeneous and complex, which hinders the development of effective treatment methods for depressive patients [8]. Therefore, it is necessary to seek appropriate nursing measures besides treatment in order to prevent depression or delay its progression. The prevention requires the identification of crucial risk factors, most of which are significantly associated with depression throughout the life cycle [9]. The most suitable way to prevent common multifactorial diseases is to transfer the entire population distribution of known risk factors, because most known risk factors for depression and anxiety are family risks, and socioeconomic status and life events are difficult or impossible to change [10]. However, there is currently little research on the influence of different gender characteristics on suicide in depressive patients. Therefore, this study is to explore the effects of personality characteristics of different genders and quality of life (QOL) on risk factors for suicide in depressive patients.

## 2. Materials and Methods

### 2.1. General Information

One hundred and eighty-six depressive patients from January 2018 to March 2019 in the Department of Psychiatry of our hospital were enrolled and divided into Groups A and B based on whether they had a suicidal tendency or not. Among them, 90 in Group A had a suicidal tendency and consisted of 42 males and 48 females, while 96 in Group B had no suicidal tendency and consisted of 44 males and 52 females.

### 2.2. Inclusion and Exclusion Criteria

Inclusion criteria: all the enrolled patients were confirmed with depression [11]. Depression was diagnosed by symptoms and general practitioners. Symptoms of depression are commonly known by the SIGECAPS mnemonic: sleep disorders, anhedonia, guilt, energy deficit, concentration deficit, appetite disorder, psychomotor retardation or agitation, and suicidality. Depressed mood and anhedonia are the two cardinal symptoms of depression. Depression may manifest differently between men and women. Women with depression are more likely to report physical ailments such as headaches, myalgias, or gastrointestinal problems. They are also more likely to exhibit emotional effects such as stress and crying easily. Men with depression are more likely to report acts of aggression, anger, substance use disorder, and risky behavior. This study was approved by the Medical Ethics Committee of our hospital; the patients and their families were informed and signed the informed consent form.

Exclusion criteria include the following: minors and patients over 60 years old, patients who did not cooperate, patients with other mental disorders, and patients with serious physical illness.

### 2.3. Methods

In this study, questionnaire surveys were carried out to analyze the effects of different gender characteristics on the risk factors for suicide in depressive patients. According to clinical interviews and self-made questionnaires, the sociodemographic data and clinical characteristics of the patients in Groups A and B were collected. Hamilton Depression Scale-17 items (HAMD-17) [12] was used to assess the patients' degree of depression, Hamilton Anxiety Scale (HAMA) [13] was used to assess their degree of anxiety, and Eysenck Personality Questionnaire (EPQ) [14] was used to evaluate their personality characteristics. QOL is defined as the subjective perception of one's own well-being within a sociocultural context. The Short Form 36 Health Survey Questionnaire (SF-36) instrument provides a concise method that is primarily used to check the health status of members of the general population as well as that of patients aged ≥14 years. As it is easy to administer, it has become one of the most widely used QOL evaluation tools in the world [15]. SF-36 measures health-related subscales, including physiological function (PF), role physical (RP), vitality (VT), bodily pain (BP), general health (GH), social function (SF), emotional function (ER), and mental health (MH), with 100 points in each dimension. BP was negatively correlated with QOL, while the rest was positively correlated with it. All questionnaire surveys should be conducted under the premise of perfect corresponding quality control measures and under the responsibility system. The questionnaires were reviewed every day to ensure that there were no missing or wrong items.

## 3. Statistical Methods

SPSS 21.0 (SPSS, Inc., Chicago, IL, USA) was used for statistical analysis. Measurement data were expressed by mean ± standard deviation ($\bar{x}\pm \text{sd}$), and their comparison between groups was analyzed by *t*-test. Count data were expressed by the number of cases/percentage (*n*/%), and the chi-square test was used for their comparison between groups. Forward and backward selection and then backward selection were performed on all the variables of high-risk factors for suicide in depressive patients, on which stepwise regression was finally conducted. Next, univariate logistic regression analysis was first performed to select important variables from the related risk factors that may cause suicide, and then, the multivariate logistic regression model was used to select important independent risk factors. *P* < 0.05 indicated a statistically significant difference.

## 4. Results

### 4.1. General Information Analysis of Males and Females with a Suicide Tendency in Group A

There were differences in actual marital status, educational level, occupations, income level, and life events between different genders with a suicidal tendency (*P* < 0.05). See Table 1 for details.

### 4.2. Characteristic Analysis on the Suicide Tendency of Depressive Patients with Different Genders

There were differences in the age of onset, degree of anxiety, moral support, positive mental attitude, and independence between male depressive patients with and without a suicidal tendency (*P* < 0.05). See Table 2 for details. There were differences in the age of onset, degree of anxiety, negative life events, moral support, positive mental attitude, intimacy, psychoticism, and neuroticism between female depressive patients with and without a suicidal tendency (*P* < 0.05). See Table 3 for details.

### 4.3. Regression Analysis on Risk Factors for the Suicide Tendency of Male Depressive Patients

The age of onset, degree of anxiety, moral support, positive mental attitude, and family independence were the independent risk factors that may cause a suicidal tendency for male depressive patients. See Table 4 for details.

### 4.4. Regression Analysis on Risk Factors for the Suicide Tendency of Female Depressive Patients

The age of onset, degree of anxiety, negative life events, moral support, positive mental attitude, family intimacy, psychoticism, and neuroticism were the independent risk factors that may cause a suicidal tendency for female depressive patients. See Table 5 for details.

### 4.5. Comparison of QOL-Related Scores

There were differences between depressive patients with and without a suicidal tendency in terms of their PF, RP, BP, SF, and ER scores (*P* < 0.05), not in GH, VT, and MH scores (*P* > 0.05). See Table 6 for details.

### 4.6. Multivariate Analysis on Risk Factors for QOL

Suicide risk factors related to QOL were selected for multivariate conditional logistic regression analysis. The results showed that low PF, RP, BP, SF, and ER may be independent risk factors for suicide in depressive patients. See Tables 7 and 8 for details.

## 5. Discussion

Depression is considered a chronic disease. The likelihood of recurrence increases with the number of episodes, often calling for prolonged maintenance of medication. Depression represents a major social and economic health issue and affects more than 350 million people worldwide, related to shortened life expectancy. It is also a major risk factor for suicide, which mainly causes deaths among young people in developed countries [16]. Suicide is the final product of complex interactions among personal health, behavioral health, and environmental factors [17]. It is estimated that there are 800,000 people committing suicides and approximately 16 million having the attempt to commit suicide worldwide every year [18]. Suicide risks depend not only on potential psychosis but also on its risk factors [19], which are various and include a series of biological, psychiatric, social-psychological, and cultural risk factors. Depressive patients with different genders may have different causes of suicide.

According to reports, males officially diagnosed with depression are less than females, and the depression incidence among males is half of that among females [20], with more common suicide attempts among females. In this study, most female depressive patients with a suicidal tendency had a low income, a large number of divorces, a low educational level, more negative events, and low family intimacy. According to previous studies, attempted suicide mostly occurs in females and unemployed and married persons [21]. Females, a younger age, and the possibility of multiple suicides are associated with a greater risk of adverse outcomes [22]. Younger and underweight females have a higher risk of depression, and well-educated and wealthy participants have a lower risk [23]. It is speculated that patients with a younger age and a lower educational level may find it more difficult to deal with their negative emotions, thus leading to their desperate situation. After experiencing negative life events, difficulties in emotional self-regulation may result in the risk of depression; there is indeed evidence that depressive patients show more frequent maladaptive strategies when regulating their emotions and have difficulties in effectively implementing adaptative strategies [24]. Additionally, female patients have neurotic personality characteristics, which indicate enhanced sensitivity, enlarged senses, and more anxiety. This suggests that we can enhance our learning ability and learn self-regulation when preventing or controlling depression progression. We can also enhance the intimacy with family members and communicate with them and friends, to gain emotional support.

In our study, male depressive patients were mostly introverted, unwilling to express their feelings, and had less social support, so they were lonelier and more unwilling to seek social help. Other studies have shown that the risk factors for males to commit suicide are possibly their MH problems, unhelpful masculinity composed of strong beliefs, social isolation, the use of other nonsocial coping strategies, life pressure, income decline, and debts [25]. Therefore, when controlling the development of depression, male patients can obtain psychological support through the somatosensory of cognitive movement and from a trustworthy and respected individual, so as to enhance their self-confidence, which may control the depression development in male patients who want to commit suicide.

This study also analyzed the QOL of patients. The results showed that patients with a suicidal tendency had lower QOL and worse physical conditions than those without suicidal tendency and that the continuous reduction of living condition may be the risk factor for the suicide. As reported before, compared with the nonsuicide group, depressive patients with a suicidal tendency have more severe depression, more complications, worse functional status, more despair, more insomnia, worse self-harm, and poorer family function [26]. This indicates that the living condition and QOL of depressive patients can be improved when their suicidal tendencies are controlled. More evidences from population studies and clinical trials show that dietary patterns and specific dietary factors may cause people to suffer from depression [27], revealing that family members can interfere with the dietary patterns of depressive patients and take them out to find their favorite foods, so as to enhance their happiness and satisfaction. Physical exercise is an effective intervention measure for depression, and its combination with antidepressants may also be a feasible adjuvant therapy [28]. This suggests that the patients can increase appropriate exercise to strengthen their constitution, RP and GH. In order to enhance their SF and ER, the family members can also take them out to participate in meaningful social activities and public service activities and then increase their social participation and presence. All of these have a positive impact on depressive patients, thus supporting them to face the disease with a positive attitude.

However, some limitations are needed to be addressed. The study was limited to a small number of participants with a recorded diagnosis of depression; a large number of populations should be performed. Meanwhile, long-term follow-up should be performed. Future studies could gain further understanding of the barriers to diagnosis by identifying participants living with depression symptoms that do not have a recorded diagnosis.

## Figures and Tables

**Table 1:** General information analysis of males and females with a suicide tendency in Group A (*n* (%)) (*x* ± sd.).

	Male (*n* = 42)	Female (*n* = 48)	*χ* ^2^/*t* value	*P* value
Age (years)	32.68 ± 5.39	34.42 ± 6.34	1.392	0.167
Course of disease (years)	2.15 ± 1.32	2.56 ± 1.21	1.537	0.127
HAMD scores	29.57 ± 3.58	30.42 ± 3.69	1/105	0.272
HAMA scores	20.73 ± 5.29	21.56 ± 5.84	0.702	0.484
Marital status			7.764	0.020
Married	25 (59.53)	14 (29.17)		
Unmarried	12 (28.57)	18 (37.50)		
Divorced or widowed	5 (11.90)	16 (33.33)		
Years of schooling (years)			15.432	≤0.001
≤9	16 (38.10)	27 (56.25)		
9-12	12 (28.57)	19 (39.58)		
≥13	14 (33.33)	2 (4.17)		
Occupations			4.742	0.029
At work	32 (76.19)	26 (54.17)		
Out of work	10 (23.81)	22 (45.83)		
Income as a proportion of family income			8.955	0.011
<40%	10 (23.81)	18 (37.50)		
40-70%	14 (33.33)	23 (47.92)		
>70%	18 (42.86)	7 (14.58)		
Negative life events before illness			5.070	0.024
Yes	24 (57.14)	38 (79.17)		
No	18 (42.86)	10 (20.83)		

Note: HAMD-17: Hamilton Depression Scale-17 items; HAMA: Hamilton Anxiety Scale.

**Table 2:** Analysis on the suicide tendency of male depressive patients.

Male	With a suicidal tendency (*n* = 42)	Without suicidal tendency (*n* = 44)	*χ* ^2^/*t* value	*P* value
Age of onset (years)	29.47 ± 3.68	36.38 ± 4.72	7.547	<0.001
HAMD-17 scores	33.41 ± 3.58	32.23 ± 3.43	1.561	0.122
HAMA scores	24.26 ± 5.24	19.63 ± 4.37	4.458	<0.001
Negative life events			0.881	0.347
Yes	28 (66.67)	25 (56.82)		
No	14 (33.33)	19 (43.18)		
Material support			0.392	0.531
Yes	22 (52.38)	26 (59.09)		
No	20 (47.62)	18 (40.91)		
Moral support			6.664	0.009
Yes	16 (38.10)	29 (65.91)		
No	26 (61.90)	15 (34.09)		
Positive mental attitude			6.768	0.009
Yes	14 (33.33)	27 (61.36)		
No	28 (66.67)	17 (38.64)		
Psychoticism	9.48 ± 2.13	8.93 ± 2.24	1.166	0.247
Neuroticism	15.20 ± 3.51	14.46 ± 2.68	1.102	0.273
Independence	5.68 ± 1.58	4.11 ± 1.42	4.851	<0.001
Contradiction	3.57 ± 1.42	3.42 ± 1.74	0.436	0.663
Intimacy	5.13 ± 2.22	5.79 ± 2.16	1.397	0.166

Note: HAMD-17: Hamilton Depression Scale-17 items; HAMA: Hamilton Anxiety Scale.

**Table 3:** Analysis on the suicide tendency of female depressive patients.

Female	With a suicidal tendency (*n* = 48)	Without suicidal tendency (*n* = 52)	*χ* ^2^/*t* value	*P* value
Age of onset (years)	26.24 ± 4.68	35.54 ± 5.23	9.341	<0.001
HAMD-17 scores	30.54 ± 4.22	29.76 ± 4.21	0.924	0.357
HAMA scores	25.31 ± 3.69	22.43 ± 3.15	4.208	<0.001
Negative life events			5.200	0.022
Yes	33 (68.75)	24 (46.15)		
No	15 (31.25)	28 (53.85)		
Material support			1.375	0.240
Yes	25 (52.08)	21 (40.38)		
No	23 (47.92)	31 (59.62)		
Moral support			3.425	0.064
Yes	17 (35.42)	28 (53.85)		
No	31 (64.58)	24 (46.15)		
Positive mental attitude			5.343	0.020
Yes	14 (29.17)	27 (51.92)		
No	34 (70.83)	25 (48.08)		
Psychoticism	8.43 ± 2.58	7.15 ± 2.34	2.602	0.010
Neuroticism	14.35 ± 3.14	12.68 ± 2.69	2.863	0.005
Independence	4.24 ± 1.58	4.41 ± 1.43	0.564	0.573
Contradiction	4.63 ± 1.67	4.46 ± 1.39	0.554	0.580
Intimacy	5.83 ± 2.14	4.62 ± 1.64	3.188	0.001

Note: HAMD-17: Hamilton Depression Scale-17 items; HAMA: Hamilton Anxiety Scale.

**Table 4:** Regression analysis on risk factors for the suicide tendency of male depressive patients.

Factors	*β*	SE	Wald	*P*	Exp (*β*)	95% CI
Age of onset	-0.266	0.131	4.047	0.044	0.634	0.594-0.991
Degree of anxiety	0.316	0.140	7.203	0.006	1.753	1.618-6.904
Moral support	-0.355	0.142	6.523	0.012	0.724	0.532-0.923
Positive mental attitude	-0.142	0.053	6.545	0.010	0.815	0.778-0.969
Independence	0.723	0.264	7.431	0.007	1.271	1.231-3.478

**Table 5:** Regression analysis on risk factors for the suicide tendency of female depressive patients.

Factors	*β*	SE	Wald	*P*	Exp (*β*)	95% CI
Age of onset	0.362	0.113	10.466	0.002	1.163	1.154-1.788
Degree of anxiety	0.191	0.066	8.422	0.005	1.152	1.062-1.371
Negative life events	0.135	0.068	3.973	0.045	1.201	1.003-1.307
Moral support	-2.013	0.876	5.288	0.021	0.256	0.021-0.715
Positive mental attitude	-1.871	0.662	7.954	0.005	0.184	0.041-0.573
Intimacy	0.194	0.081	5.779	0.015	1.075	1.046-1.429
Psychoticism	0.586	0.418	2.318	0.004	2.482	0.824-4.023
Neuroticism	0.846	0.251	11.523	0.002	1.854	1.436-3.829

**Table 6:** Comparison of QOL-related scores.

	Group A (*n* = 90)	Group B (*n* = 96)	*t* value	*P* value
PF	45.91 ± 5.69	64.28 ± 7.31	19.040	<0.001
RP	48.29 ± 4.43	57.16 ± 5.28	12.370	<0.001
BP	41.58 ± 5.29	25.29 ± 3.12	25.770	<0.001
GH	53.43 ± 4.87	54.28 ± 4.59	1.225	0.222
VT	56.27 ± 7.33	58.13 ± 6.65	1.814	0.071
SF	62.52 ± 5.56	71.75 ± 6.21	10.650	<0.001
ER	51.48 ± 3.24	60.17 ± 4.62	13.340	<0.001
MH	65.89 ± 4.61	67.17 ± 4.45	1.927	0.055

Note: QOL: quality of life; PF: physiological function; RP: role physical; VT: vitality; BP: bodily pain; GH: general health; SF: social function; ER: emotional function; MH: mental health.

**Table 7:** Main research factors and variable assignment.

Research factors	Assignment description
PF	High = 0; low = 1
RP	High = 0; low = 1
BP	Low = 0; high = 1
SF	High = 0; low = 1
ER	High = 0; low = 1

Note: PF: physiological function; RP: role physical; BP: bodily pain; SF: social function; ER: emotional function.

**Table 8:** Multivariate logistic analysis on QOL of suicide risk factors in depressive patients.

Factors	*β*	SE	Wald	*P*	Exp (*β*)	95% CI
PF	0.792	0.241	10.975	0.001	1.532	1.383-3.547
RP	2.661	0.740	12.883	≤0.001	3.604	3.344-6.483
BP	0.906	0.311	7.804	0.005	2.585	1.438-4.640
SF	1.108	0.407	6.809	0.007	1.975	1.341-7.048
ER	0.915	0.346	7.043	0.008	2.794	1.274-4.908

Note: QOL: quality of life; PF: physiological function; RP: role physical; BP: bodily pain; SF: social function; ER: emotional function.

## Data Availability

The authors confirm that the data supporting the findings of this study are available within the article.
